RETRACTED

# Triple Reassortant Swine Influenza A (H3N2) Virus in Waterfowl

**DOI:** 10.3201/eid1604.091583

**Published:** 2010-04

**Authors:** Muthannan A. Ramakrishnan, Ping Wang, Martha Abin, My Yang, Sagar M. Goyal, Marie R. Gramer, Patrick Redig, Monte W. Fuhrman, Srinand Sreevatsan

**Affiliations:** University of Minnesota, St. Paul, Minnesota, USA (M.A. Ramakrishnan, P. Wang, M. Abin, M. Yang, S.M. Goyal, M.R. Gramer, P. Redig, S. Sreevatsan); Sioux Nation Agriculture Center of Sioux Falls, Sioux Falls, South Dakota, USA (M.W. Fuhrman)

**Keywords:** Influenza A virus, triple reassortant, H3N2, waterfowl, interspecies transmission, viruses, letter

**To the Editor:** In 1998, a new lineage of triple reassortant influenza A (H3N2) virus (TR-H3N2) with genes from humans (hemmaglutinin [HA], neuraminidase [NA], and polymerase basic 1 [PB1]), swine (matrix [M], nonstructural [NS], and nucleoprotein [NP]), and birds (polymerase acidic [PA] and PB2) emerged in the U.S. swine population. Subsequently, similar viruses were isolated from turkeys (*1*,*2*), minks, and humans in the United States and Canada (*3*,*4*). In 2007, our national influenza surveillance resulted in isolation of 4 swine-like TR-H3N2 viruses from migratory waterfowl (3 from mallards [*Anas platyrrhynchos*] and 1 from a northern pintail [*Anas acuta*] of 266 birds sampled) in north-central South Dakota. We report on the characterization of these TR-H3N2 viruses and hypothesize about their potential for interspecies transmission.

Two of these isolates, A/mallard/South Dakota/Sg-00125/2007 (H3N2) and A/northern pintail/South Dakota/Sg-00126/2007 (H3N2), were recovered from the birds sampled in north-central South Dakota, 45°44′30′′N, 98°16′30′′W; 2 isolates, A/mallard/South Dakota/Sg-00127/2007(H3N2) and A/mallard/South Dakota/Sg-00128/2007(H3N2), were sampled at 45°46′30′′N, 98°15′30′′W. Viral RNA was extracted, reverse transcribed, and amplified; all segments were sequenced in entirety and submitted to GenBank under the identified virus names. Phylogenetic analysis showed significant nucleotide identities (99%–100%), differing only in 4 nucleotide positions: 1 each from PB1, PA, NP, and NS genes. Among 4 substitutions, 3 were nonsynonymous (PA, NP, and NS), and 1 (PB1) was synonymous. A1725G substitution in PB1 was identified in 2 isolates. C419T change was identified in 3 isolates (Sg-00125, Sg-00126, and Sg-00128), resulting in substitution of threonine by phenylalanine. Three isolates (Sg-00125, Sg-00126, and Sg-00127) carried an A at residue 149 of the NP gene (leading to S50N change) and 1 isolate (Sg-00128) had a G at that position (encoding serine). G809A change was present in the NP gene of 3 isolates (Sg-00125, Sg-00127, and Sg-00128). Genomes of the 4 isolates had high nucleotide and amino acid identities (>98%) with North American swine TR-H3N2 virus (A/swine/Iowa/533/99 [H3N2]). Phylogenetic analysis indicated that TR-H3N2 waterfowl and North American TR-H3N2 swine isolates belonged to a single cluster. The H3N2 subtypes from avian and swine isolates of our sequencing projects belonged to different clusters (Figure). Deduced amino acid sequences of all segments showed that these virus isolates shared common themes in virulence determinants to those previously reported for swine-like TR-H3N2 viruses (*5*).

RETRACTED

**Figure:** Phylogenetic analysis of hemagglutinin (HA) sequences from waterfowl strains isolated in this study (boldface), based on the HA gene sequences. The evolutionary associations were inferred in MEGA4.0 (www.megasoftware.net) by using the neighbor-joining algorithm with the Kimura 2-parameter gamma model and 1,000 bootstrap replications (shown on branch bifurcations). A) Evolutionary distances of waterfowl isolates from swine and avian HA (H3) sequences from the Minnesota Center of Excellence for Influenza Research and Surveillance (MCEIRS) sequencing project or Minnesota Veterinary Diagnostic Laboratory (D-Lab) database. B) Phylogeny of 230 strains, including Eurasian and North American lineages of influenza A (H3N2) viruses. Data suggest swine influenza virus (H3N2) ancestry in the waterfowl strains. GenBank accession numbers are shown. Scale bars indicate nucleotide substitutions per site.

Inasmuch as we identified a swine lineage virus in waterfowl, we first investigated laboratory contamination by using trace back and history of swine virus isolations during the time the surveillance samples were processed. No H3N2 subtype were isolated from swine sources in the Minnesota Veterinary Diagnostic Laboratory during this period. Furthermore, phylogenetic analysis of all HA segment sequences from isolates obtained in that 4-month period confirmed no contamination. We then investigated whether an ecologic niche existed for potential exposure of waterfowl to pigs. We identified a swine herd near the wildlife refuge area where the waterfowl sampling occurred. Pigs were housed outdoors, and the owner of this swine herd reported that geese and ducks inhabit the water ponds/stock dams/slough area to which the pigs had access. Contact with the local veterinarian and the South Dakota Veterinary Diagnostic Laboratory indicated no recent reports of influenza A (H3N2) episodes in the swine herd. In addition, this herd was not vaccinated for swine influenza.

The mode of transmission of swine-origin virus to waterfowl is not clear. In previously published cases, where swine influenza viruses have been identified in turkeys, the flocks were in close proximity to swine herds (*2*). Similarly, we identified a swine herd in north-central South Dakota where all 4 waterfowl were sampled. Respiratory secretions from the pigs possibly could have spread to birds through aerosols or droplets. It is also likely that swine and waterfowl shared common water sources, which contained feces from influenza-infected waterfowl or respiratory secretions from influenza-infected swine. This mode of influenza virus transmission from birds to pigs has been documented (*6*–*9*). Indeed, a waterborne source for transmission is most likely because influenza A virus can persist in water for several months depending on environmental factors such as pH, temperature, and salinity (*10*). Finally, because the swine herd in this area was housed outdoors in open pens, direct interaction with waterfowl was possible.

RETRACTED

In late 2008, serum samples were collected from this swine herd. Hemagglutination inhibition test (*1*) showed that 10 of 19 samples reacted with all 4 waterfowl isolates; titers ranged from 10 to >640. Although low titers may have occurred because pigs were exposed to heterologous cross-reactive viruses, the high titers in most animals with positive serum samples suggest exposure to an influenza (H3N2) virus similar to that recovered from the waterfowl. Our data emphasize the need to investigate the possible role of waterfowl in the maintenance and transmission of influenza A viruses to humans and to lower mammalian species.

## References

[1] Gramer MR, Lee JH, Choi YK, Goyal SM, Joo HS. Serologic and genetic characterization of North American H3N2 swine influenza A viruses. Can J Vet Res. 2007;3:2016.PMC189986617695595

[2] Tang Y, Lee CW, Zhang Y, Senne DA, Dearth R, Byrum B, Isolation and characterization of H3N2 influenza A virus from turkeys. Avian Dis. 2005;49:207–13. 10.1637/7288-101304R16094824

[3] Olsen CW. The emergence of novel swine influenza viruses in North America. Virus Res. 2002;85:199–210. 10.1016/S0168-1702(02)00027-812034486

[4] Olsen CW, Karasin AI, Carman S, Li Y, Bastien N, Ojkic D, Triple reassortant H3N2 influenza A viruses, Canada, 2005. Emerg Infect Dis. 2006;12:1132–5.1683683410.3201/eid1207.060268PMC3291069

[5] Yassine HM, Al-Natour MQ, Lee CW, Saif YM. Interspecies and intraspecies transmission of triple reassortant H3N2 influenza A viruses. Virol J. 2007;4:129. 10.1186/1743-422X-4-12918045494PMC2228287

[6] Karasin AI, Brown IH, Carman S, Olsen CW. Isolation and characterization of H4N6 avian influenza viruses from pigs with pneumonia in Canada. J Virol. 2000;74:9322–7. 10.1128/JVI.74.19.9322-9327.200010982381PMC102133

RETRACTED

[7] Karasin AI, West K, Carman S, Olsen CW. Characterization of avian H3N3 and H1N1 influenza A viruses isolated from pigs in Canada. J Clin Microbiol. 2004;42:4349–54. 10.1128/JCM.42.9.4349-4354.200415365042PMC516286

[8] Ma W, Vincent AL, Gramer MR, Brockwell CB, Lager KM, Janke BH, Identification of H2N3 influenza A viruses from swine in the United States. Proc Natl Acad Sci U S A. 2007;104:20949–54. 10.1073/pnas.071028610418093945PMC2409247

[9] Olsen CW, Karasin A, Erickson G. Characterization of a swine-like reassortant H1N2 influenza virus isolated from a wild duck in the United States. Virus Res. 2003;93:115–21. 10.1016/S0168-1702(03)00073-X12727349

[10] Brown JD, Goekjian G, Poulson R, Valeika S, Stallknecht DE. Avian influenza virus in water: infectivity is dependent on pH, salinity and temperature. Vet Microbiol. 2009;136:20–6. 10.1016/j.vetmic.2008.10.02719081209

